This article has been retracted.

# Role of Aromatherapy as a Natural Complementary and Alternative Therapy in Cardiovascular Disease: A Comprehensive Systematic Review

**DOI:** 10.1155/2022/4543078

**Published:** 2022-05-20

**Authors:** Hamdan I AlMohammed, Nada A Alanazi, Esraa Fahad Maghrabi, Manar A Alotaibi

**Affiliations:** ^1^Department of Basic Science, Faculty of Medicine, Almaarefa University, Riyadh 11597, Saudi Arabia; ^2^Faculty of Medicine, University Science Malaysia (USM), 16150 Kubang Kerian, Kelantan, Malaysia; ^3^College of Medicine, Imam Mohammad Ibn Saud Islamic University, Riyadh, Saudi Arabia

## Abstract

**Background:**

The purpose of this study was a comprehensive review of studies on the effect of aromatherapy with plant essential oils on the improvement of some conditions, for example, anxiety, stress, sleep quality, fatigue, and pain in people with cardiovascular disease.

**Materials and Methods:**

We carried out this systematic review based on the instructions of Preferred Reporting Items for Systematic Reviews and Meta-Analyses (PRISMA). Ethical agreement was not necessary as main data have not been collected. During March 2022, we searched the main English databases, for example, Google Scholar, Web of Sciences, EMBASE, EBSCO, ScienceDirect, Scopus, and PubMed/MEDLINE, with limitation to human clinical trials. For this study, no time limit was applied for the publication of articles.

**Results:**

Out of 1380 papers, 52 papers up to March 2022 were eligible for review in this systematic review. Based on the obtained results, the most widely used medicinal plants for aromatherapy in patients with cardiovascular diseases were *Lavandula angustifolia* (lavender, 55.7%), *Rosa damascena* (Damask rose, 11.5%), and *Mentha piperita* (peppermint, 5.8%), respectively. Most studies have been performed on the effect of aromatherapy on coronary angiography (21 papers, 40.4%), followed by artery bypass graft surgery (14 studies, 26.9%), and cardiac patients (5 studies, 9.6%). Most studies on the effect of aromatherapy in cardiovascular diseases were performed on anxiety (31 papers, 59.6%), sleep quality (8 studies, 15.4%), and hemodynamic parameters (6 studies, 11.5%), respectively.

**Conclusion:**

This study systematically reviewed the effects of aromatherapy in patients with cardiovascular diseases. The review of studies showed that lavender, Damask rose, and peppermint are the most frequents plants used for aromatherapy, whereas they significantly improved some illnesses and conditions, especially anxiety and sleep quality. Therefore, it can be concluded that cardiologist can used aromatherapy as a natural complementary and alternative therapy particularly with lavender, Damask rose, and peppermint to improve quality of life and some conditions such as anxiety and sleep quality.

## 1. Introduction

Cardiovascular disease (CVD), as a disease that implicates heart and blood vessels, is considered as the highest rate of morbidity and mortality worldwide [1]. Based on the World Health Organization (WHO) reports, CVD results in about 18 million deaths, which accounts for more than 30% of all global deaths [2]. Anxiety as an ambiguous and unpleasant emotion of panic can affected several aspects of human life and is considered as one of the main difficulties in people's lives [3]. Anxious patients may not be aware of the cause and source of their anxiety and may not know that the anxiety is due to a feeling of inner insecurity or is the result of an external situation in which they project their fear [3]. Today, it has been proven that stress and anxiety affect cardiovascular regulation and subsequently negatively affect cardiovascular parameters and tissue perfusion [4]. Studies in recent years continue to show that stress and anxiety can have negative effects on cortisol levels, heart rate (HR), systolic blood pressure (SBP) and diastolic blood pressure, respiratory crises, etc. [5]. In addition to cardiovascular complications, depending on the severity and duration of exposure to stress and anxiety, a person may be prone to certain diseases such as sleep disorders, neurological diseases, high blood pressure, MS, and even a weakened immune system [6]. In people with cardiovascular disease, the presence of some certain factors such as high treatment costs and poor prognosis of the disease causes stress and anxiety in patients [7]. Therefore, maintaining mental health and controlling anxiety in patients is very important.

Today, the use of synthetic drugs is no longer the best way to reduce patients' anxiety due to its many side effects. For this reason, there are many strategies, including methods available in complementary medicine, that can help control patients' anxiety [8]. One of these useful methods in complementary medicine is aromatherapy, which in recent years and in different parts of the world has received much attention compared to other complementary medicine treatments [9]. In aromatherapy, plant-derived volatile extracts and essential oils, which contain natural chemical compounds with potential medicinal effects, are used to treat diseases [10]. According to studies, during aromatherapy, plant odor, by acting on the olfactory nerve cells and subsequently activating the limbic system, can accelerate the secretion of various neurotransmitters such as enkephalin, endorphins, noradrenaline, and serotonin, and ultimately the effect. We have a reduction in patient anxiety and stress [11].

In recent years, many studies have been conducted on aromatherapy with some essential oils as a noninvasive intervention in the treatment of some diseases such as improving anxiety in patients undergoing surgery, hemodialysis, mental disorders, etc. [11, 12]. In addition to several studies, it has been shown to have a positive and therapeutic effect of aromatherapy in reducing anxiety in patients with cardiovascular disease [13]. However, a comprehensive review study about the potential effects of aromatherapy in various cardiovascular diseases such as ischemia, open heart surgery, and angiography has not yet been made, so the purpose of this study was a comprehensive review of studies on the effect of aromatherapy with plant essential oils on the improvement of some conditions, for example, anxiety, stress, sleep quality, fatigue, and pain in people with cardiovascular disease.

## 2. Materials and Methods

We carried out this systematic review based on the instructions of Preferred Reporting Items for Systematic Reviews and Meta-Analyses (PRISMA) [14]. Ethical agreement was not necessary as main data have not been collected.

### 2.1. Search Strategy

During March 2022, we searched the main English databases, for example, Google scholar, Web of Sciences, EMBASE, EBSCO, ScienceDirect, Scopus, and PubMed/MEDLINE, with limitation to human clinical trials. For this study, no time limit was applied for the publication of articles. The search strategy and keywords/MeSH terms including “Cardiovascular Diseases,” “Angiography,” “Heart Failure,” “Myocardial Ischemia,” “Heart Surgery,” “Coronary Bypass Surgery,” “Aromatherapy,” “Lavender,” “Essential Oils,” “Anxiety,” “Stress,” “Sleep Quality,” and “Blood Pressure” to find all published articles, which look at the effect of aromatherapy in patients with cardiovascular disease.

### 2.2. Selection of Studies

At first, all papers were imported into EndNote X10 (Thomson Reuters, New York, NY, USA), and duplicate publications were omitted. The titles, summary or both, of every paper were independently checked by two review authors to assess which papers should be evaluated further. The authors then examined and read full texts of all potentially eligible papers that adequately encountered the inclusion criteria for more analysis. Disagreements were resolved through consent or judged by a third review author.

### 2.3. Eligibility Criteria

In this study, the inclusion criteria of publications were as follows: full and peer-reviewed clinical trials assessing the effect of aromatherapy on patients with cardiovascular diseases were included in this study. We excluded basic experimental studies, nonclinical trial studies, studies that are presented as abstracts and only in congresses as preceding papers, and editorial papers without full text. In the next step, studies with week methodology, insufficient data, unsuitable analysis, discrepancy between methods and results, too much emphasis on important of results, and confusing presentation were excluded from this review (Figure 1).

### 2.4. Data Extraction

The extracted and required data were included authors' name (last name of first author), type of cardiovascular disease, the name of plant that was used, type of factor evaluated (e.g., anxiety, sleep quality, and hemodynamic parameters), intervention method, outcome of study, and reference.

## 3. Results

Out of 1380 papers, 52 papers up to March 2022 were eligible for review in this systematic review with the extracted required information existing in Tables 1. Based on the obtained results, the most widely used medicinal plants for aromatherapy in patients with cardiovascular diseases were *Lavandula angustifolia* (lavender, 55.7%), *Rosa damascena* (Damask rose, 11.5%), and *Mentha piperita* (peppermint, 5.8%), respectively.  Figure 2 depicted the used medicinal plants for aromatherapy in patients with cardiovascular diseases. As shown in Figure 3, most studies have been performed on the effect of aromatherapy on coronary angiography (21 papers, 40.4%), followed by artery bypass graft surgery (14 studies, 26.9%), and cardiac patients (5 studies, 9.6%). Most studies on the effect of aromatherapy in cardiovascular diseases were performed on anxiety (31 papers, 59.6%), sleep quality (8 studies, 15.4%), and hemodynamic parameters (6 studies, 11.5%), respectively (Figure 4).

## 4. Discussion

From last centuries, aromatherapy as a natural complementary and alternative therapy has been broadly used for treating various diseases and conditions [10]. In recent years, aromatherapy, which uses essential oils, has taken more attention due to its high efficacy, popularity, and extensive use. [65]. Essential oils as highly concentrated products derived from various parts of plants (e.g., leaves, root, and flowers) are composed of phytochemicals such as phenols, terpene, aldehydes, and esters, which can provide characteristic odors [66]. The external application and inhalation of oils are the main basics of aromatherapy for treating a number of mental disorders and illnesses [67]. Previous studies have been proven the promising effects of aromatherapy for improving anxiety, stress, depression, pain, sleep quality, and life quality in individuals with long-term health complications like dementia [68, 69].

Although several studies have been reported the positive and therapeutic effect of aromatherapy in patients with cardiovascular disease, a comprehensive review about the potential effects of aromatherapy in various cardiovascular diseases such as ischemia, open heart surgery, and angiography has not yet been made, so the aim of this study was to review the systematic review and determine the effects of aromatherapy with herbs. It is different in cardiovascular patients.

Out of 1380 papers, 52 papers up to March 2022, were eligible for review in this systematic review. Based on the obtained results, the most widely used medicinal plants for aromatherapy in patients with cardiovascular diseases were lavender, Damask rose, and peppermint, respectively. Most studies have been performed on the effect of aromatherapy on coronary angiography (40.4%), followed by artery bypass graft surgery (26.9%), and cardiac patients (9.6%). Most studies on the effect of aromatherapy in cardiovascular diseases were performed on anxiety (59.6%), sleep quality (15.4%), and hemodynamic parameters (11.5%), respectively.

Todays, Lavandula angustifolia Miller (lavender) is considered as one of the most frequent essential oils for treatments of mental disorders, for example, anxiety, insomnia, stress, and depression [70]. Reviews regarding the mechanisms of lavender in aromatherapy, previous studies have revealed that this plant due to the high content of terpenoid compounds such as linalool and linalyl acetate displayed their promising effects in aromatherapy for improving anxiety, and depression through some mechanisms, for example, interact with the N-methyl-D-aspartate (NMDA) receptors and dysfunction of voltage-gated calcium channels, inhibit serotonin transporter (SERT), and increased parasympathetic tone [71]. In addition, previous investigations showed that linalool and linalyl acetate as the main compounds of lavender essential oil had potent sedative effects through affecting the *γ*-aminobutyric acid type A (GABAA) receptors, indicating the promising effects of lavender essential oil on improving of sleep quality in people [72].

Rosa damascena Mill (Damask rose) belonging to the Rosaceae family is one of the most frequent aromatic herbs with various pharmacological properties in traditional and modern medicine [73]. Reviews showed that aromatherapy with Damask rose had positive effects on improving some conditions and disorders, for example, pain, anxiety, and sleep quality in various diseases such as cardiovascular ones [74]. Concerning the mechanisms of action aromatherapy with Damask rose essential oil, studies showed that this essential oil due to having some flavonoid components, nonadecane, henicosane, and docosane provokes the olfactory system, promotes parasympathetic activity, releases of endorphin and encephalin neurotransmitters, decreases the sympathetic activity, and releases cortisol and noradrenalin subsequently [75].

Another plant used in aromatherapy in cardiovascular patients is the *Mentha piperita,* which also called peppermint. Reviews showed that this plant has various pharmacological properties, for example, anxiolytic, analgesic, sedative, and sleep quality enhancer [76]. Recent clinical trials reported the potent effects of peppermint in aromatherapy for treating some illness and conditions such as anxiety, fatigue, stress, depression, and pain through affecting the olfactory pathways of the brain, decrease anxiety, relieve pain, relaxation increase, regulating pulse rate, and improving sleep quality [77]. Although studies reported the possible mechanisms of plant essential oils in aromatherapy, more studies are required to elucidate the main mechanism in various pathways [78].

## 5. Conclusion

This study systematically reviewed the effects of aromatherapy in patients with cardiovascular diseases. The review of studies showed that lavender, Damask rose, and peppermint are the most frequents plants used for aromatherapy, whereas they significantly improved some illnesses and conditions, especially anxiety and sleep quality. Therefore, it can be concluded that cardiologist can used aromatherapy as a natural complementary and alternative therapy particularly with lavender, Damask rose, and peppermint to improve quality of life and some conditions such as anxiety and sleep quality.

## Figures and Tables

**Figure 1:** Study flowchart of the current review investigation.

**Figure 2:** Frequency of the used medicinal plants for aromatherapy in patients with cardiovascular diseases.

**Figure 3:** Frequency of various cardiovascular diseases in studying the effect of aromatherapy on them.

**Figure 4:** Frequency of factors on which the effect of aromatherapy in cardiovascular diseases patients has been investigated.

**Table 1:** List of studies about the effect of aromatherapy on cardiovascular diseases.

Authors	Cardiovascular disease	Plant	Factor	Intervention	Outcome	Reference
Aalami et al.	Acute coronary syndrome	*Matricaria recutita* and neroli (6 : 2 : 0.5)	Sleep quality	Three consecutive nights	Hybrid aromatherapy caused a significant improvement in the sleep quality in patients with the acute coronary syndrome.	[15]
Abdi et al.	Coronary angiography	Orange essence	Anxiety	Two drops for 20 minutes	Aromatherapy with orange essence declined the anxiety levels after coronary angiography by 36.26 ± 7.65.	[16]
Asgari et al.	Coronary angiography	Bitter orange	Sleep quality	Two to three deep breaths	Aromatherapy with bitter orange essential oil significantly improved the sleep quality	[17]
Babatabar Darzi et al.	Artery bypass graft surgery	Lavender and damask rose	Surgical site pain severity, extubation time, and anxiety	Two drops after triggering of the first inspiration	Followed by the aromatherapy with lavender and rose essential oil, a significant reduction was observed in the time of extubation time, pain severity, and anxiety level in patients.	[18]
Bikmoradi et al	Artery bypass graft surgery	Lavender	Anxiety	Two drops for 20 minutes on the second and third days after surgery	Lavender aromatherapy had no significant effect on decreasing mental stress where it improved the systolic blood pressure.	[19]
Bikmoradi et al.	Coronary angiography	Damask rose	Anxiety	Five drops for 20 minutes	Followed by aromatherapy with damask rose essential oil, a significant decline was reported in the anxiety level.	[20]
Cho et al.	Coronary angiography	Lavender, *M. recutita,* and neroli essential oil	Anxiety, vital signs, and sleep quality	Two drops for 10 deep breaths, before and after PCI	After hybrid aromatherapy with lavender, *M. recutita*, and neroli essential oil caused a significant reduction in the anxiety level, whereas it improved the vital signs and sleep quality in undergoing coronary angiography.	[21]
Davari et al.	Artery bypass graft surgery	Lavender	Sleep Quality and Physiological Indicators	For 10 hours	Although the lavender aromatherapy had no significant effect on in the physiological indicators, it significantly improved the quality sleep in coronary artery bypass graft patients.	[22]
Ebrahimi Hosein Abadi	Artery bypass graft surgery	Lavender	Hemodynamic Indices	5 drops for 30 minutes after surgery	Lavender aromatherapy as five drops for 30 minutes after surgery improved the patient's blood pressure.	[23]
Emami-Sigaroudi et al.	Artery bypass graft surgery	Lavender and damask rose	Sleep quality	Two drops every night for 5 consecutive nights at 22 : 00.	Although aromatherapy caused an improvement in the duration, efficiency, and disturbances of sleep, no significant alteration was observed compared with the control group.	[24]
Fazlollahpour-Rokni et al. Rose	Artery bypass graft surgery	Damask rose	Anxiety	Three drops for 10 minutes one night and one hour before surgery	Aromatherapy of artery bypass graft surgery patients with Damask rose essential oil significantly declined the anxiety level.	[25]
Ganjloo et al.	Myocardial infarction	Lavender	Anxiety	Three drops for 20–30 min, 3 times a day for 3 days	Lavender aromatherapy in patients with myocardial infarction considerably reduced the overt and covert anxiety in the patient	[26]
Hajibagheri et al.	Cardiac patients	Damask rose	Sleep quality	Three drops for three subsequent nights	The sleep quality of patients was considerably improved followed by aromatherapy with damask rose essential oil.	[27]
Hasanzadeh et al.	Artery bypass graft surgery	Lavender	Anxiety	1–2 drops for 20 minutes	Lavender aromatherapy results in a considerable decrease in anxiety levels and pain intensity in patients.	[28]
Hasanzadeh et al.	Heart failure	Lavender	Fatigue	Three drops for 15 days	Lavender aromatherapy significantly improved the fatigue severity in the patients with heart failure.	[29]
Heidari et al.	Artery bypass graft surgery	Lavender	Anxiety	Two drops for 20 minutes	Lavender aromatherapy declined the anxiety score by 54.73.	[30]
Heidari Gorji et al.	Artery bypass graft surgery	Lavender	Pain perception intensity	Two drops 15 minutes	Lavender aromatherapy significantly induced the pain perception intensity on the 30 and 60-minute phases after intervention.	[31]
Hosseini et al.	Artery bypass graft surgery	Lavender	Anxiety	Two drops for 20 minutes	Lavender aromatherapy significantly decreased the anxiety and plasma cortisol levels.	[32]
Jodaki et al.	Cardiac patients	Damask rose	Anxiety and sleep quality	Five drops for three consecutive nights	After aromatherapy with Damask rose essential oil a five drops for three consecutive nights, a significant improvement in the sleep quality and anxiety level was observed.	[33]
Karadag et al.	Patients in coronary ICU	Lavender	Anxiety	Two drops for 2% essential oil, for 15 nights	Aromatherapy significantly reduced the anxiety level in the patients in coronary ICU.	[34]
Kim et al.	Coronary angiography	Lavender, Bergamot, and ylang-ylang	Anxiety, state of sleep, and satisfaction of sleep	Three drops for 5 minutes	After aromatherapy with combination of bergamot, lavender and ylang-ylang reduced anxiety levels by 39% and improved sleep satisfaction.	[35]
Koohestani et al.	Coronary angiography	Peppermint oil	Anxiety	0.2 ml for 20 minutes	Peppermint oil aromatherapy in patient candidates for angiography significantly declined the level of anxiety from 51.9 ± 5.12 to 47.9 in comparison with the control group.	[36]
Maghami et al.	Artery bypass graft surgery	Peppermint	Nausea and vomiting	Two drops 30 min before tracheal extubation, 4 h, and 8 h after endotracheal tube removal.	After aromatherapy with peppermint essential oil a significant reduction was observed in nausea and vomiting after open heart surgery.	[37]
Mahdavikian et al.	Cardiac patients	Lavender and peppermint	Fatigue	Three drops for 7 nights.	Lavender and peppermint aromatherapy significantly improved the fatigue severity in the cardiac patients.	[38]
Mirbastegan et al.	Myocardial infarction	Lavender	Anxiety	Three drops for 30 min 3 times a day for 3 days	Lavender aromatherapy in patients with myocardial infarction considerably declined the anxiety level.	[39]
Moeini et al.	Cardiac ischemia	Lavender	Sleep quality	Three nights, each time 9 hours	Followed by lavender aromatherapy, the sleep quality was significantly improved in the ischemic heart disease patients.	[40]
Moradi et al.	Cardiac ischemia	Lavender	Anxiety	Two drop for 20 min during the second and third day of hospitalization	In patients with cardiac ischemia, lavender aromatherapy considerably declined the anxiety level in comparison with the control group.	[41]
Moradi et al.	Coronary angiography	Bitter orange	Anxiety	Four ml for 15–20 minutes	Significantly improved the hemodynamic parameters and also declined the anxiety level.	[42]
Najafi et al.	Myocardial infarction	Lavender	Anxiety	Three drops for 20 min twice a day for two days	Lavender aromatherapy in patients with myocardial infarction considerably declined the anxiety level.	[43]
Nematollahi et al.	Acute coronary syndrome	Lavender, *M. recutita*, and neroli (6 : 2 : 0.5)	Anxiety	For three consecutive nights at 21 : 00 p.m.	Aromatherapy with mixture of lavender, M. recutita, and neroli (6 : 2 : 0.5) results in a significant reduction in the anxiety level in patients with the acute coronary syndrome.	[44]
Otaghi et al.	Coronary angiography	Lavender	Sleep quality	15 drops for 24 hours, every 8 hours	Lavender aromatherapy had no significant effect on the sleep quality in patients undergoing coronary angiography when compared with the control group.	[45]
Panjalizadeh B	Coronary angiography	Lavender	Anxiety	Five drops for 5 min 12 hours and 30 minutes before angiography	Lavender aromatherapy results in no considerable effect on decreasing anxiety in coronary angiography patients.	[46]
Patsalis et al.	Cardiac patients	Lavender	Anxiety	Three drops 30 min	Lavender aromatherapy in the cardiovascular patients considerably declined the anxiety level.	[47]
Pourmirzaie et al.	Coronary angiography	Lavender	Hemodynamic indexes	Two drops for 20 minutes	Followed by lavender aromatherapy a significant decrease in the hemodynamic parameters (e.g., blood pressure and respiratory rate) was observed.	[48]
Pourmovahed et al.	Artery bypass graft surgery	Lavender	Anxiety	Two drops for 20 minutes	Lavender extract aromatherapy considerably declined the level of anxiety from 45.71 to 39.53.	[49]
Rafi et al.	Coronary angiography	Lavender	Sleep quality	15 drops for 24 h before intervention	After lavender aromatherapy, a significant improvement in the sleep quality was observed in patients undergoing coronary angiography.	[50]
Rajai et al.	Artery bypass graft surgery	Lavender	Anxiety	Two drops on the morning of surgery	A considerable reduction was observed in the anxiety level (7.23 to 6.80) and heart rate followed by lavender aromatherapy with lavender.	[51]
Rambod et al.	Myocardial infarction	Lemon	Blood pressure and heart rate	Five drops for 5 minutes	Significantly improved the heart rate and anxiety on the 4th day after the intervention	[52]
Seifi et al.	Artery bypass graft surgery	Lavender	Anxiety	Two drops for 20 minutes on the second and third days after surgery	Lavender aromatherapy results in no considerable effect on decreasing anxiety in patients.	[53]
Shirzadegan et al.	Acute myocardial infarction	Geranium aroma	Anxiety	20 min a day on two consecutive days.	A considerable reduction was observed in the anxiety level.	[54]
Soleimani et al.	Cardiac patients	Peppermint	Anxiety	100% peppermint essential oil for 1 h	After aromatherapy with peppermint essential oil, a considerable decline was observed in anxiety level in cardiac patients in emergency department, when compared with the control group.	[55]
Song et al.	Coronary angiography	Lavender, ylang-ylang, and neroli oil	Stress and blood pressure	Three drops for deep breaths	Hybrid aromatherapy with lavender, ylang-ylang, and neroli oil. Results in a significant reduction in stress score and systolic blood pressure.	[56]
Tahmasebi et al.	Coronary angiography	Lavender	Anxiety	Two drops for 3 minutes	Aromatherapy caused a significant reduction in the anxiety level of patients.	[57]
Tahmasebi et al.	Coronary angiography	Lavender	Anxiety and systolic blood pressure, pulse rate, and respiratory rate	Three drops for 3 minutes	Followed by aromatherapy, a significant improvement in the anxiety and hemodynamic, and physiologic parameters was observed.	[58]
Tahmasebi et al.	Coronary angiography	Lavender	Vital sign	Three drops for 3 minutes	After aromatherapy with lavender, a significant reduction was observed in the pulse number, respiratory rate, and the systolic and diastolic blood pressure.	[59]
Tazakori et al.	Coronary angiography	Damask rose	Anxiety	15 drops for 3 times every 8 hours	Significantly improved the hemodynamic parameters and also declined the anxiety level.	[60]
Teymouri et al.	Coronary angiography	Lavender	Anxiety	Two drops for 20 minutes	Followed by the lavender aromatherapy, the level of anxiety and stress scores was significantly declined by 30.7 and 9.6, respectively.	[61]
Veiskaramian et al.	Acute coronary syndrome	Melissa	Stress	Two drops, 10–90 nights	Followed by aromatherapy with Melissa essential oil, a considerable decline was observed in stress level, arterial pressure, and heart rate 5 min after aromatherapy.	[62]
Ziyaeifard et al.	Coronary angiography	Lavender	Anxiety	Five drops for 5 min	In coronary angiography patients, lavender aromatherapy results in a significant reduction in the anxiety level	[63]
Ziyaeifard et al.	Coronary angiography	Lavender	Anxiety and pain	Five drops for 5 minutes	After aromatherapy with lavender extract, the level of anxiety was considerably reduced.	[64]
Ziyaeifard et al.	Coronary angiography	Lavender	Blood pressure and heart rate	Five drops for 5 minutes	Lavender aromatherapy caused a significant reduction in the systolic and diastolic blood pressure from as well as the heart rate after angiography.	[63]

## Data Availability

All data generated or analyzed during this study are included in this published article.
